The article "Erythrocyte-mimicking paclitaxel nanoparticles for improving biodistributions of hydrophobic drugs to enhance antitumor efficacy" was published in 2020. Journal: Drug Deliv.

# Erythrocyte-mimicking paclitaxel nanoparticles for improving biodistributions of hydrophobic drugs to enhance antitumor efficacy

**DOI:** 10.1080/10717544.2020.1731862

**Published:** 2020-02-25

**Authors:** Zheng Zhai, Pengcheng Xu, Jun Yao, Ridong Li, Lidong Gong, Yuxin Yin, Zhiqiang Lin

**Affiliations:** a Institute of Systems Biomedicine, Beijing Key Laboratory of Tumor Systems Biology, School of Basic Medical Sciences, Peking University Health Science Center, Beijing, China;; b School of Pharmacy, Inner Mongolia Medical University, Inner Mongolia, China;; c Henan Key Laboratory of Cancer Epigenetics, Cancer Institute, The First Affiliated Hospital, and College of Clinical Medicine of Henan University of Science and Technology, Luoyang, China

**Keywords:** Drug delivery, nanoparticles, biomimetic, erythrocyte membrane, paclitaxel

## Abstract

Recent decades have witnessed several nanocrystal-based hydrophobic drug formulations because of their excellent performance in improving drug loading and controlling drug release as mediate drug forms in tablets or capsules. However, the intravenous administration of drug nanocrystals was usually hampered by their hydrophobic surface properties, causing short half-life time in circulation and low drug distribution in tumor. Here, we proposed to enclose nanocrystals (NC) of hydrophobic drug, such as paclitaxel (PTX) into erythrocyte membrane (EM). By a series of formulation optimizations, spherical PTX nanoparticles (PN) with the particle size of around 280 nm were successfully cloaked in erythrocyte membrane, resulting in a PTX-NP-EM (PNM) system. The PNM could achieve high drug loading of PTX (>60%) and stabilize the particle size significantly compared to PN alone. Besides, the fluorescence-labeling PNM presented better tumor cell uptake, stronger cytotoxicity, and higher drug accumulation in tumor compared to PN. Finally, the PNM was found to be the most effective against tumor growth among all PTX formulations in tumor-bearing mice models, with much lower system toxicity than control formulation. In general, the PNM system with high drug-loading as well as superior bio-distributions *in vivo* could be served as a promising formulation.

## 1. Introduction

With the unique physicochemical properties and nanoscale effects, nanoparticle-based delivery systems have extensively been developed for a wide range of applications in drug delivery, disease imaging, and tissue engineering (Petros & DeSimone, 2010). For cancer chemotherapy, nano-delivery systems hold great potential to increase hydrophobic drug solubility and stability, achieve the effect of long-circulation as well as improve drug biodistributions for enhancing therapeutic efficacy while reducing side effects (Bjornmalm et al., 2017; Shi et al., 2017). Because of these obvious advantages of nanoparticles, a great number of clinically-available chemodrugs, including paclitaxel (PTX) (Zhang et al., 2013; Wang et al., 2017), have been formulated into various drug-loading nanoparticles to overcome the drawbacks of chemodrugs in physicochemical properties (Bernabeu et al., 2017). However, further clinical translations of nano-formulations were usually encumbered by insufficient drug loading, incomplete drug release at tumor site, low drug delivery efficiency and carrier-related toxicities (Liu et al., 2011; Sofias et al., 2017).

The article "Erythrocyte-mimicking paclitaxel nanoparticles for improving biodistributions of hydrophobic drugs to enhance antitumor efficacy" was published in 2020. Journal: Drug Deliv.

During the past two decades, there has been an explosive growth in the number of carrier-free hydrophobic drug nanocrystals available on the market or under clinical research due to their outstanding features in high drug loading as well as excellent drug release performance (Junyaprasert & Morakul, 2015; Raghava Srivalli & Mishra, 2016; Gigliobianco et al., 2018). Typically, such nanocrystals or nanosuspensions were viewed as ‘pure particles of drugs’ with a small amount or even free of surfactants. In our previous work, we found that water-insoluble drug nanocrystals markedly improved the capability of *in situ* thermosensitive gel in drug loading and drug release (Lin et al., 2014, 2015, 2016). By reviewing the nanocrystal-related products approved by the Food and Drug Administration, vast majority of drug nanocrystals were integrated into tablets or capsules as an intermediate form (Wang et al., 2012; Moschwitzer, 2013; Pawar et al., 2014; Zhang et al., 2019). Nevertheless, the intravenous administration of drug nanocrystals was usually hampered by their hydrophobic surface properties, causing short circulation time and poor bio-distribution profiles (Lu et al., 2016).

To prolong the lifetime of hydrophobic drug nanocrystals in circulation, surface modification of nanocrystals was considered to be a feasible strategy to escape immune clearance, thus achieving long-circulation effect *in vivo* to enhance drug distributions at the tumor site. Many efforts were paid in developing PEGylated drug nanocrystals to prevent them from capturing by reticuloendothelial system (RES) (Zhang et al., 2015; Luo et al., 2016; Yin et al., 2016). Despite effectiveness by such ‘escaping’ strategy at the first injection, these PEGylated particles may induce production of anti-PEG antibodies, triggering a rapid clearance of nanoparticles in circulation after repeated administrations, namely ‘accelerated blood clearance’ (ABC) phenomenon (Wu et al., 2017). Therefore, the immunogenicity of hydrophobic drug nanocrystals needs to be further reduced.

The article "Erythrocyte-mimicking paclitaxel nanoparticles for improving biodistributions of hydrophobic drugs to enhance antitumor efficacy" was published in 2020. Journal: Drug Deliv.

As an emerging platform, biomimetic cell membrane-coating technologies have intensively been developed in recent years because of their capability in disguising nanoparticles as intrinsic component, thus significantly improving pharmacokinetic properties of nanoparticles in blood circulation (Sun et al., 2017). Owing to the membrane proteins and surface glycosyl groups, erythrocyte membrane cloaking could prolong drug circulation time, escape RES uptake and reduce immunorecognition of nanoparticles (Rao et al., 2016). Furthermore, such long-circulation effect together with enhanced permeability and retention (EPR) effect of nanoparticles allowed erythrocyte-mimicking systems to carry more drugs into the tumor site (Villa et al., 2016; Fang et al., 2018). Despite the significant improvement of such camouflage-based strategy in drug delivery efficiency, cell membrane drug delivery systems were often lack of enough drug loading amount, restricting the drug dose delivered to tumor site (Han et al., 2018).

To take advantage of both technologies, we hypothesized that a cell membrane cloaking system with insoluble drug nanocrystals (NC) can achieve high drug loading, improve thermodynamic stability of NC, extend drug circulation time, improve drug accumulations in tumor, and ultimately enhance the therapeutically efficacy (Figure 1(A)).

**Figure 1.** Schematic diagram of an erythrocyte-mimicking combination nanosystem for high-dose chemotherapy. (A) *In vivo* distributions of the PNM system. The PNM is capable of delivering high-dose chemodrugs to tumor site due to high drug-loading amount of nanocrystals and high drug delivery efficiency of EM, which can disguise the nanocrystals in blood circulation system and escape from reticuloendothelial system (RES) to achieve long circulation EPR effect. (B) The components of PNM. The PNM consists of three compositions: PTX nanoparticle as solid core, PEG-PTX for hydrophilicity/hydrophobicity adjustment and biomimetic shell of erythrocyte membrane-derived vesicles.

Considering the compatibility between hydrophobic surface of paclitaxel nanoparticle and aqueous phase inside the lipid bilayer of erythrocyte membrane (EM), polyethyleneglycol-conjugated paclitaxel (PEG-PTX), an amphiphilic molecule, was synthesized as an intermediate layer for preparation of a PTX-NP-EM (PNM) system (Figure 1(B)). The PNM consisted of three components. The first component was solid drug core (PN) with extremely high drug loading. Different from typical polymeric nanoparticles, hydrophobic drug nanocrystals were regarded as ‘pure drug particles’ with drug loading efficiency up to 100%. The drugs in PN existed in the form of crystal instead of drug molecules in polymeric nanoparticles (Rabinow, 2004). The second component was intermediate hydration layer (PEG-PTX) for hydrophilicity/hydrophobicity adjustment. As an amphiphilic molecule, PEG-PTX was terminated with the hydrophobic PTX molecule, enabling it embedded into PN structure. The other segment of PEG made the surface of PN more hydrophilic, thus enhancing its flexibility with EM. The third component was erythrocyte-mimicking shell (EM), derived from endogenous red blood cells. EM could disguise PN from endocytosis of macrophages, thus carrying more drugs into tumor site due to the EPR effect (Figure 1(B)). Following a similar protocol, DiR, a near infrared dye, was used to prepare PTX/DiR hybrid NP-EM (PDNM) for fluorescence labeling of the PNM. Subsequently, these formulations were further investigated in terms of *in vitro* characterization, cellular uptake, cytotoxicity, biodistributions and antitumor efficacy as well as preliminary safety evaluations to test our hypothesis.

The article "Erythrocyte-mimicking paclitaxel nanoparticles for improving biodistributions of hydrophobic drugs to enhance antitumor efficacy" was published in 2020. Journal: Drug Deliv.

## 2. Materials and methods

### 2.1. Materials

Paclitaxel (>99% purity) was purchased from Dalian Meilun Biotechnology Co. (Dalian, China). Pluronic^®^ F127, Polyethylene glycol (mPEG_2000_) and Cremophor EL^®^ were purchased from Sigma-Aldrich Co. (St. Louis, MO). 4-Dimethylaminopyridine (DMAP) and Succinic anhydride were bought from Energy Chemical Co. (Shanghai, China). Diisopropylethylamine (DIEA) and 1-ethyl-3-(3-dimethyllaminopropyl) carbodiimide hydrochloride (EDCI) were obtained from Innochem Co. (Beijing, China). 1,1-dioctadecyl-3,3,3,3-tetramethylindotricarbocyanine iodide (DiR) was acquired from AAT Bioquest Inc. (Sunnyvale, CA). All the analytical reagent grade solvents for synthesis were purchased from Tong Guang fine chemical Inc. (Beijing, China). HPLC grade methanol and acetonitrile were obtained from Thermo Fisher Scientific Co. (Local Agent in Shanghai, China). Unless stated otherwise, all chemicals were used without purification.

Dulbecco’s modified Eagle’s medium (DMEM) and penicillin/streptomycin for cell culture were purchased from Corning Co. (Corning, NY). Fetal bovine serum (FBS) was provided by Gibco, Invitrogen Corp. (Carlsbad, CA). Cell lines including 4T1, 3T3, MCF-7, 293 T, HT29, HepG2, and MDA-MB-486 were obtained from American Type Culture Collection (ATCC) (Manassas, VA). All the cell lines were cultured in DMEM supplemented with 10% FBS and 1% antibiotics at 37 °C in 5% CO_2_ humidified atmosphere. Female BALB/c mice (22–25 g) were purchased from the Vital Laboratory Animal Center (Beijing, China) and kept under specific-pathogen-free (SPF) condition for 1 week before studies. All animal experiments were approved by Animal Care and Use Committee of Peking University Health Science Center.

The article "Erythrocyte-mimicking paclitaxel nanoparticles for improving biodistributions of hydrophobic drugs to enhance antitumor efficacy" was published in 2020. Journal: Drug Deliv.

### 2.2. Synthesis of mPEG_2000_-PTX conjugates (PEG-PTX)

PEG-PTX was synthesized according to a previously reported method (Zhang et al., 2015). Firstly, mPEG_2000_ (4 g, 2 mmol) and succinic anhydride (1 g, 10 mmol) were stirred in the solvent of toluene (50 ml) and pyridine (2 ml) under reflux. 24 h later, 100 ml of water was added to quench the reaction. Then, the solution was extracted via ethyl acetate (50 ml) for three times, washed with brine and evaporated to remove the solvent. The resulting intermediate mPEG_2000_-COCH_2_CH_2_COOH was collected. Next, mPEG_2000_-COCH_2_CH_2_COOH (2.1 g, 1 mmol) was mixed with EDCI (384 mg, 2 mmol), DIEA (0.33 ml, 2 mmol) and DMAP (12 mg, 0.1 mmol) in CH_2_Cl_2_ (20 ml) under ice bath for 30 min. After that, PTX (852 mg, 1 mmol) was added under magnetic stirring and maintained at room temperature for 24 h. The reactant was concentrated and purified by column chromatography on silica gel (CH_2_Cl_2_:CH_3_OH = 10:1) to obtain the mPEG_2000_-PTX. All the above reactions were monitored by thin layer chromatography constantly. The final product of PEGylated PTX was characterized by ^1 ^H-NMR.

### 2.3. Preparation of PTX nanoparticles (PNs)

To delicately control the shape and size of the nanoparticles, we prepared the PNs according to a modified protocol in previous literature (Lin et al., 2015). Specifically, Rod-shaped PNs were produced through film dispersion method and subsequent incubation-sonication procedure. Briefly, PTX (1 mg) together with F127 (5 mg) were first dissolved in CH_2_Cl_2_ (0.5 ml) followed by nitrogen blowing and 30 min vacuum drying to form a thin layer of film. After 40 min hydration and 10 min vortex, the samples were sonicated with 0.9% saline for 15 min to obtain the PN suspension.

Spherical-shaped PNs with various particle sizes were prepared by the method of emulsion-lyophilized crystallization (Ni et al., 2015). Firstly, PTX and F127 at various concentrations and ratios were dissolved in CH_2_Cl_2_. Then the solution was added to deionized water (20 ml) under the conditions of probe sonication (Sonics Vibra cell, VCX 750) with amplitude of 30% for 10 min. Then, the resulting emulsion was immediately frozen in liquid nitrogen for further lyophilization. Finally, the lyophilized powder was dissolved in deionized water and centrifuged at the speed of 200,000 *g* for 60 min. The final precipitation was resuspended to obtain pure PN with spherical shape.

### 2.4. Preparation of PEG-PTX/PTX (PEGylated PN), PTX/DiR (PDN), PEG-PTX/PTX/DiR (PEGylated PDN) hybrid nanoparticles

mPEG_2000_-PTX was used to formulate PEGylated hybrid PN following a similar protocol in the section of 2.3. Briefly, different ratio of PEG-PTX and PTX (30:1-3:1 w/w) together with F127 were solved in CH_2_Cl_2._ After that, the solution was added to DI water via probe sonication, lyophilization, centrifugation and resuspension to obtain PEGylated PN.

The article "Erythrocyte-mimicking paclitaxel nanoparticles for improving biodistributions of hydrophobic drugs to enhance antitumor efficacy" was published in 2020. Journal: Drug Deliv.

The fluorescence labeling of nanoparticles was achieved by incorporating DiR in nanoparticles. The PDN and PEGylated PDN were prepared following the same protocol as described above for PN and PEGylated PDN except addition of DiR in CH_2_Cl_2_ together with PTX (PTX: DiR = 10:1 w/w).

### 2.5. Extraction of erythrocyte membranes

The preparation of red blood cell (RBC) ghosts and removal of hemoglobin contents were performed following previously protocols (Chai et al., 2017). Heparinized fresh whole blood was first collected from female BALB/c mice (22–25 g) and then centrifuged at the speed of 1000 *g* for 5 min at 4 °C to carefully devoid the serum and buffy coat. The separated red blood cells were washed by precooled phosphate buffer saline (PBS) before hemolysis in hypotonic medium (0.25 × PBS, pH = 5.8 with protease inhibitor cocktails) for 20 min. Then, the lysate was centrifuged at 1000 *g* for 5 min to remove the hemoglobin. The resulting centrifugal residues were further suspended in 0.9% saline as purified RBC membrane.

### 2.6. Preparation of erythrocyte membrane-derived vesicles and encapsulation of nanoparticles

The solution of the murine RBC ghost was sonicated for 10 min and extruded through 400 nm polycarbonate porous membranes for 9 times by an Avanti mini extruder to form erythrocyte membrane-derived vesicles. To prepare EM-clocking nanoparticles, PEGylated PN or PDN was mixed with the above vesicles via sonication for 10 min, respectively. For full encapsulation by EM, 1 mg of PTX hybrid nanoparticles were mixed well with EM vesicles extracted from 1 ml of whole blood. This ratio was estimated based on the volume of erythrocyte and surface area of nanoparticles reported beforehand (Chai et al., 2017).

### 2.7. *In vitro* characterization of various nanoformulations

The particle size and zeta potential of the freshly prepared nanoformulations were measured by dynamic light scattering (DLS) analysis using a Malvern Zetasizer Nano ZS (Malvern, U.K.) at 25 °C. The morphology of the nanoformulations was observed by transmission electron microscopy (TEM, JEOL, JEM-1400, Japan). To prepare samples for TEM observation, different nanoformulations were deposited on copper nets with supporting film for 90 s, followed by negative staining with 1% uranyl acetate for another 90 s.

The article "Erythrocyte-mimicking paclitaxel nanoparticles for improving biodistributions of hydrophobic drugs to enhance antitumor efficacy" was published in 2020. Journal: Drug Deliv.

### 2.8. Protein characterization of the PNM and erythrocyte membranes vesicles

To analyze the protein content of nanoparticles, samples of PN, PEGylated PN, the PNM and RBC ghost were boiled in SDS loading buffer, which were then run on a 10% SDS-PAGE gel together with protein marker for electrophoresis separation (Bio-Rad, Mini-PROTEAN^®^Tetra). The resulting gel was stained by Coomassie Blue to visualize the protein bands.

### 2.9. *In vitro* stability of PN, PEGylated PN, and the PNM

The physical stability of various nanoformulations was evaluated on the basis of the change of appearance and particle size. Briefly, freshly prepared samples were stored in separate test tubes at 4 °C. At determined time points over 8 days, each sample was taken some photographs by a digital camera followed by particle size analysis. Prior to size determination, samples were vortexed for 1 min.

### 2.10. Drug loading amount of PN, PEGylated PN, and the PNM

The drug loading efficiency of each nanoformulation was determined by high performance liquid chromatography with ultraviolet detector (HPLC-UV) (Thermo Scientific UltiMate 3000). Briefly, PN, PEGylated PN or the PNM were divided into two equal portions, respectively. One was dissolved and diluted in methanol and subsequently injected into HPLC system through C18 column (Thermo Scientific, Hypersil GOLD™, 250 × 4.6 mm) and eluted by mobile phase (acetonitrile/water, 60/40, v/v). The wavelength of UV detector was set at 231 nm. The amount of PTX in various nanoformulations was calculated from a standard curve. The other one was lyophilized into powders whose weight was indicated as the total amount of corresponding nanoformulation. The percentage of drug loading for each formulation was calculated by the formula as follows: Drug loading (%) = the amount of PTX in each formulation/total amount of each formulation.

### 2.11. *In vitro* leakage and release studies

*In vitro* drug leakage and release behavior of different formulations including PN, Taxol^®^ and the PNM were investigated by the dialysis method (Lin et al., 2014). Briefly, various formulations containing 1 mg of PTX were sealed in pre-swollen dialysis bags (Cutoff = 12,000–14,000 Da) and immersed into 50 ml of medium (DMEM medium with 10% FBS for drug leakage experiments or 1.0 M sodium salicylate solution for drug release experiments) at 37 °C, followed by shaking at the speed of 40 rpm. At each time point, 20 μl of medium was withdrawn and replaced with an equal volume of fresh medium. Then, the withdrawn medium was diluted with 40 μl of acetonitrile prior to injection into an HPLC system for the detection of PTX concentrations. The analysis conditions were the same as in Section 2.10.

The article "Erythrocyte-mimicking paclitaxel nanoparticles for improving biodistributions of hydrophobic drugs to enhance antitumor efficacy" was published in 2020. Journal: Drug Deliv.

### 2.12. Verification of DiR hybrid nanoparticles (PDN)

To verify formation of PTX/DiR hybrid nanoparticles, a series of experiments were performed. Firstly, PDN suspensions were imaged by a NIR imaging system (PerkinElmer, Lumina XR, λex = 720 nm, λem = 790 nm) to confirm imaging capacity of DiR in the PDN system. Then, PDN suspensions were separated into three portions after centrifugation at 4000 rpm as follows: (1) Precipitate. The precipitate at the bottom was collected; (2) Residue. The supernatant was subsequently filtrated through a 50-nm membrane to obtain residue on the membrane; (3) Flitrate. The filtrate was also collected after membrane filtration of supernatant. Finally, the above three samples together with original PDN were diluted by 10-fold methanol and imaged using a Lumina XR system, respectively. The fluorescence intensities of all samples were quantified by fluorospectrophotometry. The relative fluorescence value of original PDN via methanol dilution was considered as 100% and those of the other samples were recorded as corresponding percentages.

### 2.13. Cellular uptake study

To study cellular uptake of various nanoparticles, we performed near infrared imaging on cells incubated with the DiR formulations. Briefly, six cell lines including 293 T, HT29, HepG2, MDA-MB-486, MCF-7, 4T1 were seeded into a 24-well plate at the density of 10^5^ cells/well. After 80–90% confluence, the cells were incubated with various fluorescent formulations (free DiR, PDN and the PDNM) containing equal levels of DiR for 2 h. Treatment with PBS was used as a negative control. Subsequently, the cells in each well were washed with precooled PBS for three times and imaged by Lumina XR imaging system (PerkinElmer, IVIS Lumina, Waltham, MA).

### 2.14. *In vitro* cytotoxicity of PTX formulations

To measure *in vitro* cytotoxicity of different PTX formulations (PN, PEGylated PN and the PNM), we conducted an MTS assay (CellTiter 96^®^AQ_ueous_ Non-Radioactive Cell Proliferation Assay, Promega) against 4T1 cells and 3T3 cells following the manufacturer’s instructions (Zhai et al., 2019). Briefly, cells were seeded in 96-well plates at the density of 5000 cells per well. After 12-hour incubation, various concentrations of nano-formulations were added and incubated for 48 h. Then, 20 μl of MTS solution was mixed with the medium in each well followed by determination of absorbance at 490 nm in a microplate reader (Flexstation 3). Finally, the cell viability curves for each formulation were plotted and the relevant IC_50_ values were calculated from triplicate experimental data.

### 2.15. *In vivo* imaging of PDN and the PDNM

Female BALB/c mice (6–8 weeks) were subcutaneously inoculated with 4T1 cells (10^6^) under the right armpit. When tumor size reached about 50 mm^3^, each 4T1-bearing mouse received an intravenous injection of PDN or the PDNM at dose of 31 μg/kg DiR, respectively. At predetermined time points (hour 1, 4, 8, 12, and 24) post administration, each mouse was anesthetized with 2% isoflurane via a nose cone and imaged by a Lumina XR imaging system. After 24 h living imaging, mice were sacrificed by cervical dislocation for collection of tumors and main organs including heart, liver, spleen, lung, and kidney which were further imaged by the same imaging system. Excitation and emission wavelength were set at 780 nm and 845 nm, respectively.

The article "Erythrocyte-mimicking paclitaxel nanoparticles for improving biodistributions of hydrophobic drugs to enhance antitumor efficacy" was published in 2020. Journal: Drug Deliv.

### 2.16. *In vivo* pharmacodynamic and preliminary safety studies of PN and the PNM

The 4T1-xenografted BALB/c mice models were developed for *in vivo* pharmacodynamic and preliminary safety studies. 4T1 cells (10^6^) were inoculated under the right armpits of the mice. When tumor size reached about 200 mm^3^ after one week, mice were randomly assigned into 3 groups (*n* = 5) for intravenous injections of saline, PN and the PNM (10 mg/kg) every day, respectively. Tumor size and body weight of the mice were monitored using a vernier caliper and a balance at day 7, 9, 11, 14, 16, and 18. Tumor volume was calculated by following the formula: V = 1/2 × (length) × (width)^2^. On day 18, all mice were sacrificed by cervical dislocation. Tumors and main organs including heart, liver, spleen, lung, and kidney were excised, weighed and then collected for frozen sections and H&E staining. The pathological changes at histological levels were observed and analyzed under a microscope.

### 2.17. Statistical analysis

All experimental data were expressed as mean ± standard deviation (SD) and analyzed using student’s *t*-test or a one-way analysis of variance (ANOVA) with GraphPad Prism 7 software. A *p* value less than 0.05 indicated statistically significant.

## 3. Results and discussions

### 3.1. Preparation of PN, PEGylated PN, and the PNM

For successful cloaking by EM, the PNs with various surface properties were precisely prepared by different formulation technologies. Here, we explored the effect of shape, particle size and surface property of PN on membrane cloaking.

At first, we adopted previously-reported film dispersion method to produce rod-like nanocrystals by bottom-up spontaneous crystal growth (Supplementary Figure S1(A)). Due to inappropriate length–width ratio (>5), these nanoparticles failed to be encapsulated by EM in our experiments (Figure 2(A)). Then, we prepared spherical PN by emulsion solvent evaporation method (Ni et al., 2015), in which the crystal growth of PTX molecules were confined in oil-in-water (O/W) emulsion droplets at nanoscale (Supplementary Figure S1(B), Figure 2(B)). The particle size of sphere-like PN was precisely manipulated by controlling the feed ratios of PTX to F127 and the amount of solvent volume. Supplementary Table S1 lists the nanoparticles with various particle size ranging from 263.5 ± 10.36 nm to 660.0 ± 55.62 nm. Although it has been reported that nanoparticles with diameter of 65-350 nm can be coated by cell membrane, none of the above nanoparticles in Supplementary Table S1 were successfully cloaked by EM. We speculated that it was probably due to strong hydrophobicity of PN surface, making it difficult to be encapsulated into the inner water core of cell membrane with structure of phospholipid bilayers. For this reason, we then managed to improve the surface properties of PNs by PEGylation modification. To obtain PEGylated PNs, PTX conjugated with PEG (PEG-PTX) was synthesized ((Figure 2(C), Supplementary Figure S2) and verified by ^1^H NMR (Supplementary Figure S3). With the same segment, PEG-PTX was co-crystallized with PTX to form hybrid PN (PEGylated PN). By controlling the ratio of PEG-PTX to PTX, this unique method enabled us to create the PNs with varying degrees of surface hydrophilicity. As shown in Supplementary Table S2, higher percentage of PEG-PTX resulted in larger PEGylated PNs with wider polymer dispersity index (PDI). All the PEGylated paclitaxel nanoparticles were able to be cloaked by EM, suggesting that the PEGylation is necessary for cell membrane coating. Theoretically, introduction of PEG-PTX has the detrimental effect for PTX to exert its cytotoxicity due to the steric hindrance of PEG chains. However, low-density PEGylation by 5% of PEG-PTX has little influence on cytotoxicity of PTX-NC in a previous report (Zhang et al., 2015). Therefore, the PNM with the least ratio of PEG-PTX to PEG (1:30, <5%) was chosen for subsequent studies.

The article "Erythrocyte-mimicking paclitaxel nanoparticles for improving biodistributions of hydrophobic drugs to enhance antitumor efficacy" was published in 2020. Journal: Drug Deliv.

**Figure 2.** *In vitro* characterization of PN, PEGylated PN, and the PNM. (A) and (B) showed the morphology of nod-shaped PN and spherical-shaped PN by TEM, respectively; (C) and (D) represented particle size distribution of PEGylated PN and the PNM, respectively, measured by DLS and TEM; (E) Comparison of average particle size of PN, PEGylated PN, and the PNM; (F) Zeta potential of PN, PEGylated PN, and the PNM; (G) SDS-PAGE gel analysis of protein content in PN, PEGylated PN, and the PNM referred to RBC lysate; the error bars indicated ± SD (*n* = 3).

Based on the above exploration of formulations, the successfully prepared PNM were composed of three layers with distinctive functions (Figure 1(B)). The innermost layer was a solid drug core, namely PN, which could offer extremely high drug loading levels for sufficient dose delivered to tumor site. The intermediate layer was amphiphilic PEG-PTX for adjustment the surface of PN to enhance its flexibility with EM. The outermost layer was erythrocyte-mimicking shell (EM) for the escape of RES uptake to achieve a long-circulation effect in blood. Together with the EPR effect, the PNM were capable of delivering more drugs to the cancer site.

### 3.2. *In vitro* characterization of the PNM

After preparation optimization, we applied a series of methods for the PNM characterization *in vitro*. Transmission electron microscopy (TEM) pictures showed spherical PN and the PNM with a particle size of more than 200 nm. By comparison of their morphologies, the PNM had obvious membrane structure, providing a visible evidence for cell membrane cloaking (Figure 2(C,D)).

According to dynamic light scattering (DLS) assay, the particle size of the PNM (327.50 ± 9.54 nm) was marginally larger than that of PEGylated PN (295.53 ± 8.03 nm) and PN (277.53 ± 1.16 nm), resulting from the hydration radius of PEG chains and the thickness of cell membranes (Figure 2(E)). These results also support EM coating on the surface of nanoparticle. The size difference between PEGylated PN and the PNM exactly matched the thickness of EM at around 8-10 nm, consistent with previous literature (Kroll et al., 2017). The uniform size less than 400 nm together with low PDI value (<0.2) enabled the PNM to form stable nano-systems *in vitro*, which was crucial for drug delivery in circulation after intravenous administrations (Figure 2(C,D)).

Figure 2(F) shows that the zeta potential of the PNM reached −8.83 ± 0.51 mV, similar to the zeta potential of EM as reported (Gao et al., 2017) and significantly higher than that of PN (−1.59 ± 0.29 mV) and PEGylated PN (−2.09 ± 0.25 mV) in the level of charge values, further confirming successful EM cloaking on the surface of the PEGylated PN. Nearly neutral zeta potential of PEGylated PN made it possible for the nanoparticles to be encapsulated into negatively charged cell membranes (Hu et al., 2011; Figure 2(F)).

In blood circulation, the integrity of membrane proteins serves a critical role for erythrocyte to avoid RES uptake. Therefore, we performed SDS-PAGE analysis (Rao et al., 2017) to characterize the protein components of the PNM. As shown in Figure 2(G), the PNM retained almost all membrane proteins compared to the original erythrocyte membranes, illustrating that the preparation process of the PNM rarely affected the composition of surface proteins.

The article "Erythrocyte-mimicking paclitaxel nanoparticles for improving biodistributions of hydrophobic drugs to enhance antitumor efficacy" was published in 2020. Journal: Drug Deliv.

### 3.3. *In vitro* formulation evaluations of the PNM

Stability, drug loading, drug leakage and drug release are significant parameters for *in vitro* evaluations of a novel formulation as well as *in vivo* therapeutic effect. In this study, the stability of various nanoparticles was assessed by the phenomenon of precipitation generation during storage process (Choi and Park, 2016). Over 8 days at 4 °C, the PNM kept stable all the time while apparent aggregations and precipitations emerged for both PN and PEGylated PN (Figure 3(A)). Similarly, DLS assay indicated that the particle size of PN increased from 270 to 450 nm over two months, but PEGylated PN and the PNM remained constant size all the time (Figure 3(B)). This improved stability was probably ascribed to dual protection of EM shell and intermediate layer of PEG-PTX.

**Figure 3.** *In vitro* stability, drug loading and drug release properties of PN, PEGylated PN, and the PNM. (A) Digital photo of three nanoparticles storage at 4 °C taken at indicated time, visible sediments were pointed by yellow arrow; (B) Change of particle size of three nanoparticles in two months’ storage; (C) PTX loading rate of three nanoparticles determined by HPLC; (D) Drug leakage performance of formulations; (E) Cumulative percentage of drug release from various formulations; all the scale bars indicated ± SD (*n* = 3).

High drug loading efficiency is of significance to guarantee high-dose of drugs to be delivered into tumor tissue. Although a large number of nanocarriers with novel functions have been reported, it still remains a challenge for many nanoparticles to maintain high drug loading amount as well as good stability simultaneously. As indicated in Figure 3(C), the PTX loading efficiency of the PNM was over 60%, much higher than that of the other polymeric nano-systems. Therefore, the solid paclitaxel core provides high drug level for the PNM system, crucial for sufficient drugs delivered to tumor site.

Then, drug leakage tests were performed under mimic physiological conditions. As shown in Figure 3(D), both formulations maintained inert in leakage medium containing blood serum similar to body fluid components, guaranteeing their stability during the circulation. Under sink condition, relatively slow release manner was observed for PNM, with 60% cumulative drug release in two days. This is probably because cell membranes coat of PNM protects the inner PN core from dissolution (Figure 3(E)).

### 3.4. Cellular uptake and cytotoxicity studies

After *in vitro* characterization, we investigated the cellular uptake behaviour of the PNM by a fluorescence-labeling method. To label the PTX nanoparticles, DiR, a near-infrared dye, was used to formulate PTX/DiR hybrid NP (PDN), PEGylated PDN, and erythrocyte membrane coating PTX/DiR hybrid NP (PDNM) (Sharma et al., 2015). Upon incorporating DiR, the hybrid nanoparticles exhibited no obvious difference compared to the corresponding nanoparticles without DiR in particle size (Supplementary Figure S4(A,C)) and zeta potential (Supplementary Figure S4(B)). Then, an exclusion strategy by a method of fluorospectrophotometry was adopted to verify the formation and imaging capability of PTX/DiR hybrid nanoparticles (Figure 4(A)). In water dispersion system, the PDN emitted strong fluorescence compared to PN with no signals, indicating that DiR played an important role in the PDN. To further analyze the existing forms of DiR, in free dyes or hybrid state, we employed various physical methods to separate the nanoparticles and then quantitatively compare fluorescent intensities of different components via a 10-fold methanol dilution. After centrifugation, fluorescence intensity of the precipitate was only 24.8%, illustrating that the majority of DiR stayed in the solutions. Following centrifugation and filtration (cutoff = 50 nm), the fluorescence signal was mostly in residues instead of filtrates, suggesting that DiR existed primarily in nanoparticles.

The article "Erythrocyte-mimicking paclitaxel nanoparticles for improving biodistributions of hydrophobic drugs to enhance antitumor efficacy" was published in 2020. Journal: Drug Deliv.

**Figure 4.** Cellular uptake of nanoparticles with fluorescence labeling. (A) Confirmation of DiR hybrid nanoparticles. All the nanoparticles were separated by centrifuge and filtration, the fluorescence intensity was detected by resolved precipitate in solvent, which showed almost all DiR successfully hybrid into nanoparticles with only a few free DiR left in suspension; (B) Comparison of cellular uptake of PDN and PDNM on various cell lines, visualized by DiR fluorescence imagining.

Figure 4(B) shows that the PDNM emitted much stronger fluorescence signals than PDN in different cancer cells, suggesting that EM shell played an essential role in promoting cellular uptake of nanoparticles. According to previously-reported mechanisms of cellular uptake, endocytosis of the PNM would most likely be mediated by membrane fusion, resulting in increased uptake on nanoparticles by cancer cells compared to PDN (Fu et al., 2015). In contrast, incubation of DiR solution with cells showed little fluorescence. Owing to the water-insolubility, free DiR probably existed in the form of micro-scale particles, leading to difficulty in endocytosis by tumor cells (Chen & Li, 2015).

To further explore the antiproliferative activity and toxicity of formulations, we performed MTS experiments against 4T1 murine tumor cells and 3T3 murine normal cell line. In both cell lines, PEGylated PN displayed slightly lower cytotoxicity than PN. It was speculated that the PEG-modified nanoparticles may affect affinity and internalization, leading to weaker anti-proliferation activity (Arranja et al., 2016; Rao et al., 2017). In cancerous 4T1 cell line (Figure 5(A)), the PNM exhibited the strongest antitumor effect among all the formulations with reduced IC_50_ values than PN (Supplementary Table S3). However, PNM exhibited much lesser cytotoxicity than Taxol in normal cell line, such as 3T3 (Figure 5(B)), thus ensuring better selectivity and lower side effect.

The article "Erythrocyte-mimicking paclitaxel nanoparticles for improving biodistributions of hydrophobic drugs to enhance antitumor efficacy" was published in 2020. Journal: Drug Deliv.

**Figure 5.** Cytotoxicity of formulations on cell lines. (A) Cytotoxicity of formulations on 4T1 murine breast cancer cell line for 48 h incubation, * *p* < 0.05 vs PN, ** *p* < 0.01 vs PN; (B) Cytotoxicity of formulations on 3T3 murine fibroblast cell line for 48 h incubation, **p < 0.01 vs Taxol, *** *p* < 0.001 vs Taxol; error indicated ± SD (*n* = 4).

### 3.5. *In vivo* imaging of the fluorescence-labeled PNM

For *in vivo* imaging, PDN and the PDNM were administrated intravenously into 4T1 tumor-bearing BALB/c mice, which were subsequently imaged at different timepoints. From 4 to 24 h post administration, the PDNM presented much stronger fluorescence at tumor site than PDN did, suggesting the important role of EM on enhancing accumulation of nanoparticles at tumor site. Interestingly, liver signals in the PDNM group decreased more rapidly compared to that in PDN group. It was probably because of entrapment of PDN in livers while the PDNM successfully escaped from RES (Arranja et al., 2016; Figure 6(A)). These data illustrated that EM-based long circulation effect together with EPR effect by nanoparticles could achieve preferential drug accumulations in tumor tissue.

**Figure 6.** *In vivo* NIR fluorescence imaging of DiR-labeled PDN and PDNM. (A) *In vivo* imaging of 4T1 cancer-bearing BALB/c mice receiving a single injection of PDN or PDNM, respectively. The dashed black circles indicate the tumor burden. (B) *Ex vivo* imaging of tumor and organs excised from 4T1 tumor-bearing mice 24 h post injections of the two fluorescent formulations. Compared to PDN, the PDNM showed higher drug distributions at tumor site. The yellow arrows point to the tumor tissue.

For *ex vivo* imaging, mice were sacrificed for collection of main organs 24 h post injection. The fluorescence of the PDNM inside tumor was significantly higher than that of PDN group, further proving that EM-coating technology indeed enhanced drug accumulations at tumor site (Figure 6(B)). Besides tumor, the PDNM presented more fluorescence distributions in the other organs than PDN did (Figure 6(B)), likely due to the long-circulation effect of the PDNM, leading to more drug distributions at various organs.

The article "Erythrocyte-mimicking paclitaxel nanoparticles for improving biodistributions of hydrophobic drugs to enhance antitumor efficacy" was published in 2020. Journal: Drug Deliv.

### 3.7. *In vivo* antitumor pharmacodynamic studies and preliminary toxicity evaluations

After *in vivo* evaluation of the PNM, we carried out antitumor pharmacodynamic studies on 4T1-xengrafted BALB/c mouse models. Compared to control and PN group, the PNM was the most effective formulation in antitumor efficacy, benefitting from higher cellular uptake efficiency, stronger cytotoxicity and better drug accumulations at tumor site (Figure 7(A,B,D)).

**Figure 7.** *In vivo* antitumor activity of different PTX formulations against 4T1-xenografted BALB/c mice. (A) Tumor growth curve of different mouse groups with administrations of saline, PN (PTX dose 10 mg/kg) and the PNM (PTX dose 10 mg/kg); (B) Weight of *ex vivo* tumors from the mice sacrificed by cervical dislocation at the experimental end point; (C) Body weight change of mice in different groups; (D) Image of excised tumors from different groups; (E) Representative organs of mice from control group and PNM treated group, metastatic nodules of lung tissue from control group directed by yellow arrow; error bars indicated ± SD (*n* = 5 for each group), *p < 0.05, **p < 0.01.

By observation on *ex vivo* organs, we found some symptoms such as liver and spleen enlargement and even lung metastasis in control tumor-bearing mice without any drug treatment. In contrast, no tumor metastasis and gross morphological abnormalities was observed in the mice receiving injections of the PNM. It indicated that the PNM was capable of preventing tumor metastasis beyond inhibiting primary tumors, probably because potential tumor metastasis organs were also the tissues in which nanoparticles distributed preferentially (Figure 7(E)). What’s more, no significant change in body weight was observed during the treatment period for both PDN and PN group (Figure 7(C)).

### 3.8. Histological studies

To further explore the toxicities of various formulations at the histological level, we performed H&E staining on tissue sections from main organs. Despite both PN and the PNM exhibited significant antitumor activity, the PNM caused less side effects than PN did (Figure 8). Firstly, liver sections from the control group showed structural disorders of hepatic lobules and expansion of hepatocytes under inflammation while those from the PN and PNM group remained normal, suggesting that the treatment of PTX nanoparticles could relieve the liver damage on tissue level. Secondly, in consist with general observation, the control group showed widespread lung-metastasis tumor nodules, which was prevented upon PN and PNM treatment. Thirdly, myocardial damage was found in PN treated group characterized by myocardial fibrosis, local hemorrhage, and structural disorder, but the damages were mitigated in PNM group. Finally, as one of the most common adverse reactions caused by PTX, nephrotoxicity was observed in PN treated group, illustrated by renal cell edema and severely damaged nephron structure, while the toxic effects were reprieved in PNM group (Figure 8). Cardiac and renal toxicity were the mostly reported side effects of paclitaxel (Marupudi et al., 2007). PN as a pure form of paclitaxel nanoparticle inevitably caused these damages. However, under the protection of erythrocyte membrane camouflage, PNM treatment did not result in obvious cardiac and renal toxicity. Based on the above results, it could be concluded that PNM hold lower toxicity and improved safety margin.

The article "Erythrocyte-mimicking paclitaxel nanoparticles for improving biodistributions of hydrophobic drugs to enhance antitumor efficacy" was published in 2020. Journal: Drug Deliv.

**Figure 8.** H&E staining of tissue sections (40×) from different treatment groups, black arrows pointed at obvious morphological changes. The lesions in liver and metastases in lung from control group were relieved once received PN and PNM treatment. Moreover, cardiac and renal toxicities of PTX were significantly alleviated in PNM treated group compared to PN.

## 4. Conclusions

In this study, we developed a PNM system by enclosing surface-modified paclitaxel nanoparticles into erythrocyte membrane. The PNM is around 320 nm with spherical morphology, consisting of three components including solid drug core (PN), hydration layer (PEG-PTX) and biomimetic shell (EM). The PN core contributes to a high drug loading of PTX (>60%) while EM shell preserving good physical stability without precipitation for at least 8 days and constant particle size over 2 months. Moreover, the fluorescence-labeling PNM showed better cellular uptake and more drug accumulations at tumor site compared to PN using *in vivo* imaging. Accordingly, the PNM presented stronger cytotoxicity at cell levels and better antitumor efficacy in 4T1 tumor-bearing mice models, with much lower toxicity than control formulation. It can be concluded that the PNM, which disguise high drug-loading paclitaxel nanoparticles *in vivo*, may serves as an efficient delivery system for high-dose chemotherapy at tumor site.
